The article "Oxidative Stress and Its Related Factors in Latent Autoimmune Diabetes in Adults" was retracted in 2024. Reasons: signs of a paper mill; suspected computer-generated content; unreliable results or conclusions; concerns about the data.

# Oxidative Stress and Its Related Factors in Latent Autoimmune Diabetes in Adults

**DOI:** 10.1155/2021/5676363

**Published:** 2021-09-13

**Authors:** Jinjin Li, Yuan Zhang, Jingyun Zhang, Rongna Dong, Juanjuan Guo, Qiumei Zhang

**Affiliations:** ^1^NHC Key Laboratory of Hormones and Development, Tianjin Key Laboratory of Metabolic Diseases, Chu Hsien-I Memorial Hospital & Tianjin Institute of Endocrinology, Tianjin Medical University, Tianjin 300134, China; ^2^Department of Genetics, College of Basic Medical Sciences, Tianjin Medical University, Tianjin 300070, China

## Abstract

**Aims:**

Few research was reported to explore oxidative stress in individuals with latent autoimmune diabetes in adults (LADA). Therefore, our goal is to study oxidative stress and related factors in LADA patients.

**Methods:**

In this study, 250 Chinese inpatients were diagnosed with LADA (*n* = 110) and type 2 diabetes mellitus (*n* = 140) and 140 healthy volunteers were recruited. Moreover, individuals with LADA were followed for 6 months to evaluate whether short-term glycemic control during hospitalization can improve oxidative stress. Clinical and laboratory measurements of height, weight, blood pressure, glycosylated hemoglobin (HbA_1c_), blood lipids, 8-isoprostaglandin F2*α* (8-iso-PGF2*α*), and superoxide dismutase (SOD) were performed. Stepwise multiple regression analyses were used to assess factors that related to oxidative stress in individuals with LADA.

**Results:**

Compared with patients with type 2 diabetes, individuals with LADA have better oxidative stress and worse oxidative stress than healthy volunteers. After multiple regression analyses, systolic blood pressure, HbA_1c_, duration of diabetes, and diabetic retinopathy were associated with 8-iso-PGF2*α* and HbA_1c_. Diabetic retinopathy and diabetic ketosis were associated with SOD in individuals with LADA. Our results also revealed that, after 6 months of follow-up, oxidative stress was improved to some extent in persons with LADA.

**Conclusions:**

Our results show that compared with type 2 diabetes, LADA means less oxidative stress, and compared with healthy volunteers, it means more oxidative stress. Systolic blood pressure, HbA_1c_, duration of diabetes, diabetic retinopathy, and ketosis were associated with oxidative stress in individuals with LADA. Furthermore, short-term glycemic control can improve oxidative stress to some extent in individuals with LADA.

## 1. Introduction

Latent autoimmune diabetes in adults (LADA) is a kind of adult-onset autoimmune diabetes [1], which shows the features of both type 1 and type 2 diabetes mellitus. Until now, immunogenetic, clinical, and metabolic characteristics that are unique to LADA have been extensively studied [2, 3]. For example, compared with patients with type 2 diabetes, LADA patients have poorer blood sugar control and insulin deficiency [4]. However, the pathological mechanism clearly defined by LADA has not yet been fully elucidated. Thus, defining the unique characteristics of LADA helps to understand the progression of the disease and its complications, which will contribute to early prevention and treatment of the condition as well as subsequent tissue damage.

The article "Oxidative Stress and Its Related Factors in Latent Autoimmune Diabetes in Adults" was retracted in 2024. Reasons: signs of a paper mill; suspected computer-generated content; unreliable results or conclusions; concerns about the data.

Oxidative stress results from an imbalance between the generation of reactive oxygen species (ROS) and the antioxidant defense systems [5, 6]. 8-iso-PGF2*α* is one of the most abundant and well-recognized isoprostanes in human plasma and urine and is now recognized as a “gold-standard” biomarker for in vivo oxidative stress and lipid peroxidation [7–9]. Many studies [10] have observed that the stable 8-iso-PGF2*α* level in patients with type 2 diabetes is significantly higher than that of healthy people or nondiabetic patients. At the same time, people have long recognized that SOD high levels of excessive reactive oxygen species play an important role in cancer, diabetes, inflammatory diseases, and various cardiovascular diseases [11, 12]. Thus, 8-iso-PGF2*α* and SOD were selected as indicators of oxidative stress.

Many researches have reported that diabetes mellitus was associated with oxidative stress, leading to an increased production of ROS or reduction of the antioxidant defense system [13, 14]. Therefore, the balance between the free radical generating system and the free radical scavenging system is extremely important in diabetes. However, most previous studies have focused on studying the oxidative stress of type 2 diabetes [15, 16]. Recently, evidence has shown that there was also significant oxidative stress in type 1 diabetes mellitus, but the study of oxidative stress in type 1 diabetes is mostly confined to the children and animals, and few studies were reported to explore oxidative stress in LADA [15, 16]. Therefore, this study is aimed at investigating oxidative stress and its related factors in individuals with LADA, and whether short-term glycemic control during hospitalization can improve oxidative stress.

## 2. Methods

### 2.1. Study Design and Participants

This study was performed in Tianjin Metabolic Diseases Hospital, China, from January 2015 to December 2017. 250 Chinese inpatients were diagnosed with LADA (*n* = 110) and type 2 diabetes mellitus (*n* = 140), and 140 no-diabetes healthy controls were recruited. In addition, LADA patients were followed up for 6 months after discharge to assess whether short-term blood glucose control during hospitalization could improve oxidative stress. The exclusion criteria are as follows: age < 18 years; evidence of kidney, liver, or heart failure; pregnant and lactating; evidence of malignancy. All participants were provided the written informed consent, and the protocol was approved by the Human Ethics Committee of Tianjin Medical University.

The article "Oxidative Stress and Its Related Factors in Latent Autoimmune Diabetes in Adults" was retracted in 2024. Reasons: signs of a paper mill; suspected computer-generated content; unreliable results or conclusions; concerns about the data.

### 2.2. Blood Collection and Clinical Measurements

Fasting morning blood samples were collected from all participants by venous puncture into 5 mL tubes. Height and weight measurements were taken after patients took off their shoes and changed into an examination gown. Blood pressure was measured by a standard mercury sphygmomanometer with the participants seated after at least 5 minutes of rest. HbA_1c_ and lipid profiles (triglyceride, TG; high-density lipoprotein-cholesterol, HDL-C; low-density lipoprotein-cholesterol, LDL-C) were obtained from laboratory measurements. Information on GAD antibodies, diabetic complications, duration of diabetes, and medication use (antioxidant drug, antihypertension drug, etc.) were retrieved from medical records.

### 2.3. Assessment of Oxidative Stress

Enzyme-linked immunosorbent assay was used to detect the levels of 8-iso-PGF2*α*, and intra- and interassay CVs both were 15%. Water-soluble tetrazolium was used to detect the level of SOD activity, and intra- and interassay CVs were 5.05% and 3.32%, respectively.

### 2.4. Definitions of Variates

Type 2 diabetes mellitus is diagnosed according to the World Health Organization (WHO) criteria [17]. LADA is defined as the age of onset of diabetes which is 30 years or older, circulating pancreatic islet autoantibodies, and no signs or symptoms of typical type 1 diabetes [18]. Diabetic nephropathy was defined as patients with a history of diabetes, and microalbumin/creatinine > 300 mg/g, or diagnosis by the renal biopsy. All patients with primary glomerular disease and other secondary glomerular diseases were excluded.

### 2.5. Statistical Analysis

Clinical characteristics were described in all of the participants using mean and standard deviations (SD) for continuous variables and percentages for categorical variables. Continuous variables were compared by one-way analysis of variance and categorical variables by chi-squared tests. We evaluated the association between clinical biological makers and oxidative stress using Pearson's correlation for parametric variables and Spearman's rank correlation for nonparametric variables. Stepwise multiple regression analyses were used to assess factors that related to oxidative stress. All statistical analyses were performed using SPSS version 17.0. *P* values < 0.05 indicated statistical significance.

The article "Oxidative Stress and Its Related Factors in Latent Autoimmune Diabetes in Adults" was retracted in 2024. Reasons: signs of a paper mill; suspected computer-generated content; unreliable results or conclusions; concerns about the data.

## 3. Results

The mean age of the participants was 45.55 ± 8.90 years with 47% males. The characteristics of the participants are shown in Table 1. Individuals with LADA had lower body mass index, diastolic blood pressure, systolic blood pressure, LDL-C, TG, and higher HDL-C compared with type 2 diabetes, but there was no significant difference between LADA and healthy volunteers. Additionally, there was no significant difference in HbA_1c_, diabetic peripheral neuropathy, diabetic retinopathy, and macroangiopathy between LADA and type 2 diabetes.

Individuals with LADA had a decreased level of 8-iso-PGF2*α* activity compared to type 2 diabetes and an increased level of 8-iso-PGF2*α* activity compared to healthy volunteers (Figure 1(a)). In addition, compared with patients with type 2 diabetes, LADA patients have higher levels of SOD activity, while compared with healthy volunteers, SOD activity levels are lower (Figure 1(b)).

Correlation analyses between 8-iso-PGF2*α*, SOD, and clinical characteristics in individuals with LADA are shown in Table 2; systolic blood pressure, HbA_1c_, diabetic nephropathy, duration of diabetes, diabetic retinopathy, and diabetic ketosis were related to 8-iso-PGF2*α*; and HbA_1c_, diabetic nephropathy, duration of diabetes, diabetic retinopathy, and ketosis were related to SOD.

Stepwise multiple regression analyses were used to assess factors that related to oxidative stress in LADA. As shown in Table 3, after multiple regression analyses, systolic blood pressure, HbA_1c_, duration of diabetes, and diabetic retinopathy were associated with 8-iso-PGF2*α*, and HbA_1c_, diabetic retinopathy, and ketosis were associated with SOD.

Individuals with LADA were followed up for 6 months after short-term glycemic control from hospital. Our results revealed that, after 6 months of follow-up, TG, HbA_1c_, 8-iso-PGF2*α*, and SOD levels were decreased and body mass index, diastolic blood pressure, systolic blood pressure, LDL-C, and HDL-C were not significantly different in persons with LADA (Table 4).

## 4. Discussion

Our findings revealed that individuals with LADA imply less oxidative stress compared to type 2 diabetes and more oxidative stress compared to healthy volunteers. Systolic blood pressure, HbA_1c_, duration of diabetes, diabetic nephropathy, diabetic retinopathy, and ketosis were related to oxidative stress in LADA. In addition, short-term blood glucose control can improve oxidative stress in LADA patients. As far as we know, this is the first published research to examine oxidative stress in individuals with LADA.

Our results suggested that LADA implies more oxidative stress compared to healthy volunteers. Some studies have reported that diabetes mellitus was correlated with oxidative stress, leading to an increased production of ROS or reduction of the antioxidant defense system, which were in line with our study. In addition, a number of research reports claim that isoprostaglandin 8-iso-PGF2a is a clear biomarker of oxidative stress in a variety of human diseases, including immune diseases such as diabetes, cardiovascular disease, and rheumatoid arthritis [7, 19]. A cohort study among 62 diabetes patients found that diabetes mellitus was related to increased formation of 8-iso-PGF2*α* [20]. Besides, an experimental study reported the protective effect of chemically modified SOD on lipid peroxidation and antioxidant status in diabetic rats [21].

The article "Oxidative Stress and Its Related Factors in Latent Autoimmune Diabetes in Adults" was retracted in 2024. Reasons: signs of a paper mill; suspected computer-generated content; unreliable results or conclusions; concerns about the data.

Our findings also revealed that LADA implies less oxidative stress compared to type 2 diabetes. There may be several reasons to explain this phenomenon. In this study, individuals with type 2 diabetes have higher body mass index, diastolic blood pressure, systolic blood pressure, LDL-C, TG, lower HDL-C, and worse diabetic nephropathy than LADA. Firstly, elevated levels of TG and LDL-C and decreased levels of HDL-C caused elevated serum-free fatty acids. Previous studies have reported that high concentrations of free fatty acids can induce ROS production in a variety of different tissues, leading to lipotoxicity [22]. Secondly, many studies showed that increased oxidative stress was a hallmark of hypertension [23, 24]. Additionally, a study also reported that 8-iso-PGF2*α*, an oxidative stress marker, was elevated in hypertensive patients [25]. These previous findings were in line with our results that type 2 diabetes patients had a higher blood pressure and a worse oxidative stress status. Thirdly, type 2 diabetes patients have worse complications than LADA. Oxidative stress plays a pivotal role in the development of diabetes complications, both cardiovascular and microvascular [26]. A review also showed that ROS plays a central role in the development and progression of diabetic nephropathy [27]. The above factors may cause individuals with LADA to have less oxidative stress than type 2 diabetes.

This study found that short-term glycemic control during hospitalization might improve oxidative stress to some extent in individuals with LADA. Hyperglycemia is a common factor in diabetic patients. Directly generating ROS or changing the redox balance is the main contributor to oxidative stress [28]. Moreover, hyperglycemia can cause membrane lipid peroxidation and oxidative stress markers increase. In diabetic patients, blood glucose concentrations could be assessed by the HbA_1c_. A cross-section study [29], including 1527 Japanese adults, found that 8-iso-PGF2*α* was significant associated with HbA_1c_ and can be a reliable marker of impaired glucose tolerance. Imig [30] also reported that under the condition of hyperglycemic, the formation and release of 8-iso-PGF2*α* by porcine vascular smooth muscle cells were enhanced. Therefore, a good glycemic control can reduce oxidative stress and inflammatory pathway activation.

The article "Oxidative Stress and Its Related Factors in Latent Autoimmune Diabetes in Adults" was retracted in 2024. Reasons: signs of a paper mill; suspected computer-generated content; unreliable results or conclusions; concerns about the data.

Our study had strengths and limitations. A strength of our study is that it explores the oxidative stress and its related factors in LADA patients, hitherto not extensively examined. In addition, it is clear that this provides an advantage in terms of “oxidative stress” because any internally treated patients will have higher levels of oxidative stress factors during hospitalization. However, this is a cross-section study, which is impossible to infer causality. Moreover, the information on insulin, oral hypoglycemic agent status, and c-peptide were lacking, which is intrinsically related to oxidative stress and may affect our results.

## 5. Conclusion

Our findings revealed that LADA implies less oxidative stress compared to type 2 diabetes and more oxidative stress compared to healthy volunteers. In addition, short-term blood glucose control can improve the oxidative stress of LADA patients to a certain extent. Additionally, we will further conduct cohort and basic mechanism research to confirm our findings.

## Figures and Tables

**Figure 1:** Comparison of 8-iso-PGF2*α* and SOD levels in LADA, type 2 diabetes mellitus, and healthy volunteers. (a) Comparison of 8-iso-PGF2*α* levels in LADA, type 2 diabetes mellitus, and healthy volunteers. (b) Comparison of SOD levels in LADA, type 2 diabetes mellitus, and healthy volunteers. ^∗∗^*P* < 0.001.

**Table 1:** Clinical characteristics of study population during hospitalization.

Parameter	LADA	Type 2 diabetes mellitus	Healthy volunteers	*P* value^∗^
*n*	110	140	140	
Male (*n*, %)	58 (52.7)	64 (45.7)	62 (44.3)	0.10
Age (year)	44.7 ± 13.3	45.8 ± 6.8	45.9 ± 5.9	0.52
BMI (kg/m^2^)	21.4 ± 2.7	26.4 ± 3.5	21.3 ± 3.4	≤0.001
SBP (mmHg)	118.1 ± 12.9	132.0 ± 17.0	122.9 ± 20.5	≤0.001
DBP (mmHg)	72.4 ± 8.5	78.5 ± 8.5	73.3 ± 11.1	≤0.001
HbA_1c_ (mmol/mol)	74 (17)	76 (20)	34 (16)	≤0.001
HbA_1c_ (%)	8.9 ± 1.64	9.1 ± 1.8	5.2 ± 1.5	≤0.001
LDL-C (mmol/L)	2.9 ± 0.7	3.4 ± 1.2	2.9 ± 0.9	≤0.001
HDL-C (mmol/L)	1.5 ± 0.7	1.4 ± 0.4	1.5 ± 0.2	0.02
TG (mmol/L)	1.3 ± 0.9	2.5 ± 1.0	1.3 ± 0.8	≤0.001
8-iso-PGF2*α* (pg/mL)	626.8 ± 94.2	678.2 ± 95.3	528.8 ± 80.9	≤0.001
SOD (U/mL)	110.9 ± 23.0	100.4 ± 24.0	130.7 ± 21.1	≤0.001
Duration of diabetes (years)	7.3 ± 4.3	7.1 ± 5.1	—	0.68
Diabetic nephropathy (*n*, %)	17 (15.5)	55 (39.3)	—	≤0.001
Peripheral neuropathy (*n*, %)	48 (43.6)	65 (46.4)	—	0.32
Diabetic retinopathy (*n*, %)	37 (33.6)	39 (27.9)	—	0.42
Diabetic ketosis (*n*, %)	40 (36.4)	21 (15.1)	—	≤0.001
Macroangiopathy (*n*, %)	33 (30.0)	44 (31.4)	—	0.81

Abbreviations: BMI: body mass index; SBP: systolic blood pressure; DBP: diastolic blood pressure; LDL-C: low-density lipoprotein-cholesterol; TG: total triglycerides; HDL-C: high-density lipoprotein-cholesterol; LADA: latent autoimmune diabetes in adults. ^∗^*P* values < 0.05 indicated statistical significance.

The article "Oxidative Stress and Its Related Factors in Latent Autoimmune Diabetes in Adults" was retracted in 2024. Reasons: signs of a paper mill; suspected computer-generated content; unreliable results or conclusions; concerns about the data.

**Table 2:** Correlation analyses between 8-iso-PGF2*α*, SOD, and clinical characteristics in LADA patients.

Parameter	8-iso-PGF2*α*		SOD	
	*r*	*P*	*r*	*P*
BMI (kg/m^2^)	0.03	0.78	-0.02	0.81
SBP (mmHg)	0.28	≤0.001	-0.18	0.06
DBP (mmHg)	0.08	0.40	-0.06	0.55
HbA_1c_ (%)	0.59	≤0.001	-0.42	≤0.001
LDL-C (mmol/L)	0.08	0.41	-0.10	0.37
HDL-C (mmol/L)	-0.03	0.78	0.01	0.95
TG (mmol/L)	0.05	0.10	-0.11	0.27
SOD (U/mL)	-0.73	≤0.001	-0.73	≤0.001
Duration (year)	0.44	≤0.001	-0.45	≤0.001
Diabetic nephropathy	0.35	≤0.001	-0.32	≤0.001
Peripheral neuropathy	0.10	0.29	-0.15	0.11
Diabetic retinopathy	0.43	≤0.001	-0.44	≤0.001
Diabetic ketosis	0.25	0.01	-0.26	0.01
Macroangiopathy	0.06	0.46	-0.06	0.45
Diabetic nephropathy	0.35	≤0.001	-0.32	≤0.001

**Table 3:** Stepwise multiple regression analyses between clinical parameters and 8-iso-PGF2*α*, SOD in individuals with LADA.

Parameter	Nonstandardized coefficient		Standard coefficient	*t* value	*P* value
	*B*	Standard error			
*8-iso-PGF2α*					
(constant)	134.22	58.08		2.31	0.02
SBP (mmHg)	1.11	0.44	0.15	2.51	0.01
HbA_1c_ (%)	33.72	3.48	0.59	9.68	≤0.001
Duration of illness (years)	5.30	1.11	0.32	4.75	≤0.001
Diabetic nephropathy	44.97	18.43	0.17	2.43	0.02
Diabetic retinopathy	26.44	14.94	0.13	1.77	0.08
Diabetic ketosis	22.03	11.98	0.11	1.83	0.07
*SOD*					
(constant)	13.99	0.56		24.99	≤0.001
SBP (mmHg)	-0.13	0.30	-0.04	-0.45	0.66
HbA_1c_ (%)	-0.13	0.04	-0.33	-3.49	≤0.001
HDL-C (mmol/L)	-0.49	0.64	-0.08	-0.77	0.44
Diabetic retinopathy	-1.18	0.52	-0.24	-2.27	0.03
Diabetic ketosis	-1.41	0.39	-0.30	-3.64	≤0.001

**Table 4:** Changes in clinical characteristics during baseline and 6 months of follow-up in individuals with LADA.

Parameter	Baseline	Follow-up	*t* value	*P* value
BMI (kg/m^2^)	21.4 ± 2.7	21.5 ± 2.8	0.10	0.92
SBP (mmHg)	118.1 ± 12.9	117.9 ± 12.3	0.25	0.80
DBP (mmHg)	72.5 ± 8.5	72.1 ± 7.9	0.78	0.44
LDL-C (mmol/L)	2.9 ± 0.7	2.8 ± 0.6	1.32	0.19
HDL-C (mmol/L)	1.5 ± 0.7	1.5 ± 0.8	0.07	0.94
TG (mmol/L)	1.3 ± 0.9	1.3 ± 0.3	5.37	≤0.001
HbA_1c_ (mmol/mol)	74 (17)	62 (17)	4.98	≤0.001
HbA_1c_ (%)	8.9 ± 1.6	7.8 ± 1.6	4.98	≤0.001
8-iso-PGF2*α* (pg/mL)	626.8 ± 94.2	601.4 ± 75.0	2.21	0.02
SOD (U/mL)	110.9 ± 23.0	116.5 ± 40.2	2.12	0.04

The article "Oxidative Stress and Its Related Factors in Latent Autoimmune Diabetes in Adults" was retracted in 2024. Reasons: signs of a paper mill; suspected computer-generated content; unreliable results or conclusions; concerns about the data.

## Data Availability

The datasets used and analyzed during the current study can be solicited to the corresponding author or the first author.

## References

[1] Rolandsson O., Palmer J. P. (2010). Latent autoimmune diabetes in adults (LADA) is dead: long live autoimmune diabetes!. *Diabetologia*.

[2] Andersen M. K., Lundgren V., Turunen J. A. (2010). Latent autoimmune diabetes in adults differs genetically from classical type 1 diabetes diagnosed after the age of 35 years. *Diabetes Care*.

[3] Fourlanos S., Dotta F., Greenbaum C. J. (2005). Latent autoimmune diabetes in adults (LADA) should be less latent. *Diabetologia*.

[4] Andersen C. D., Bennet L., Nyström L. (2013). Worse glycaemic control in LADA patients than in those with type 2 diabetes, despite a longer time on insulin therapy. *Diabetologia*.

[5] Reuter S., Gupta S. C., Chaturvedi M. M., Aggarwal B. B. (2010). Oxidative stress, inflammation, and cancer: how are they linked?. *Free Radical Biology & Medicine*.

[6] Sinha N., Dabla P. K. (2015). Oxidative stress and antioxidants in hypertension-a current review. *Current Hypertension Reviews*.

[7] Milne G. L., Sanchez S. C., Musiek E. S., Morrow J. D. (2007). Quantification of F_2_-isoprostanes as a biomarker of oxidative stress. *Nature Protocols*.

[8] Musiek E. S., Morrow J. D. (2005). Quantification of F2-isoprostanes by gas chromatography/mass spectrometry as a measure of oxidant stress. *Current Protocols in Toxicology*.

[9] Wiswedel I. (2009). F(2)-isoprostanes: sensitive biomarkers of oxidative stress in vitro and in vivo: a gas chromatography-mass spectrometric approach. *Methods in Molecular Biology*.

[10] Costacou T., Evans R. W., Schafer G. L., Orchard T. J. (2013). Oxidative stress and response in relation to coronary artery disease in type 1 diabetes. *Diabetes Care*.

[11] Adiga I. K., Nair R. R. (2008). Multiple signaling pathways coordinately mediate reactive oxygen species dependent cardiomyocyte hypertrophy. *Cell Biochemistry and Function*.

[12] Carpagnano G. E., Lacedonia D., Palladino G. P. (2012). Could exhaled ferritin and SOD be used as markers for lung cancer and prognosis prediction purposes?. *European Journal of Clinical Investigation*.

[13] Yang H., Jin X., Kei Lam C. W., Yan S. K. (2011). Oxidative stress and diabetes mellitus. *Clinical Chemistry and Laboratory Medicine*.

[14] Sklavos M. M., Bertera S., Tse H. M. (2010). Redox modulation protects islets from transplant-related injury. *Diabetes*.

[15] Henriksen E. J., Diamond-Stanic M. K., Marchionne E. M. (2011). Oxidative stress and the etiology of insulin resistance and type 2 diabetes. *Free Radical Biology & Medicine*.

The article "Oxidative Stress and Its Related Factors in Latent Autoimmune Diabetes in Adults" was retracted in 2024. Reasons: signs of a paper mill; suspected computer-generated content; unreliable results or conclusions; concerns about the data.

[16] Asmat U., Abad K., Ismail K. (2016). Diabetes mellitus and oxidative stress--A concise review. *Saudi Pharmaceutical Journal : SPJ : the official publication of the Saudi Pharmaceutical Society*.

[17] Alberti K. G., Zimmet P. Z., WHO Consultation (1998). Definition, diagnosis and classification of diabetes mellitus and its complications. Part 1: diagnosis and classification of diabetes mellitus provisional report of a WHO consultation. *Diabetic Medicine : a journal of the British Diabetic Association*.

[18] Redondo M. J. (2013). LADA: time for a new definition. *Diabetes*.

[19] Yu G. F., Jie Y. Q., Wu A., Huang Q., Dai W. M., Fan X. F. (2013). Increased plasma 8-iso-Prostaglandin F2*α* concentration in severe human traumatic brain injury. *Clinica Chimica Acta; International Journal of Clinical Chemistry*.

[20] Schwedhelm E., Bartling A., Lenzen H. (2004). Urinary 8-iso-prostaglandin F2alpha as a risk marker in patients with coronary heart disease: a matched case-control study. *Circulation*.

[21] Mansuroglu B., Derman S., Yaba A., Kizilbey K. (2015). Protective effect of chemically modified SOD on lipid peroxidation and antioxidant status in diabetic rats. *International Journal of Biological Macromolecules*.

[22] Gerber P. A., Rutter G. A. (2017). The role of oxidative stress and hypoxia in pancreatic beta-cell dysfunction in diabetes mellitus. *Antioxidants & Redox Signaling*.

[23] Majzunova M., Dovinova I., Barancik M., Chan J. Y. (2013). Redox signaling in pathophysiology of hypertension. *Journal of Biomedical Science*.

[24] Ndisang J. F., Vannacci A., Rastogi S. (2014). Oxidative stress and inflammation in obesity, diabetes, hypertension, and related cardiometabolic complications. *Oxidative Medicine and Cellular Longevity*.

[25] de Faria A. P., Fontana V., Modolo R. (2014). Plasma 8-isoprostane levels are associated with endothelial dysfunction in resistant hypertension. *Clinica Chimica Acta; International Journal of Clinical Chemistry*.

[26] Giacco F., Brownlee M. (2010). Oxidative stress and diabetic complications. *Circulation Research*.

[27] Stanton R. C. (2011). Oxidative stress and diabetic kidney disease. *Current Diabetes Reports*.

[28] Fiorentino T. V., Prioletta A., Zuo P., Folli F. (2013). Hyperglycemia-induced oxidative stress and its role in diabetes mellitus related cardiovascular diseases. *Current Pharmaceutical Design*.

[29] Mure K., Yoshimura N., Hashimoto M. (2015). Urinary 8-iso-prostaglandin F2*α* as a marker of metabolic risks in the general Japanese population: the ROAD study. *Obesity*.

[30] Imig J. D. (2000). Eicosanoid regulation of the renal vasculature. *American Journal of Physiology-Renal Physiology*.

